The article "Diagnostic Value of Magnetic Resonance Susceptibility-Weighted Imaging Scanning in Different Types of Early Prostate Cancer" was retracted in 2023. Reasons: unreliable results or conclusions; lack of ethics approval or compliance; concerns about the data; concerns about the peer review.

# Diagnostic Value of Magnetic Resonance Susceptibility-Weighted Imaging Scanning in Different Types of Early Prostate Cancer

**DOI:** 10.1155/2022/4884646

**Published:** 2022-05-23

**Authors:** Ruihui Gao, Jiayuan Liu, Hengcheng Zhu

**Affiliations:** ^1^Department of Urology, People's Hospital, Dongxihu District, Wuhan, Hubei 430040, China; ^2^Department of Urology, Wuhan University People's Hospital, Wuhan, Hubei 430060, China

## Abstract

To investigate the cost of MRI-sensitive imaging (SWI) for early-stage prostate cancer. In 2019, the research group included a total of 60 leukemia patients, all of whom were diagnosed with prostate-specific antigen (PSA). According to the range of PSA values, they were group A (18 cases), group A 0-44 mg/ml (18 cases), and group B 4-1010 mg/ml (26 cases). 10 mg/ml was divided into C group (16 cases). Another 60 patients with benign prostatic hyperplasia treated at the same time served as a control group. All patients underwent sensitive MRI scanning, followed by diagnostic and clinical evaluation of weighted MRI scanning to diagnose various types of prostate cancer. The results showed that there was no difference in Ve levels among the three groups (*P* > 0.05); the SUSE score and Ktrans and Kep levels of the patients in group C were higher in groups B, A, and A (*P* < 0.05). In patients with early leukemia, SUSE score was significantly correlated with Ktrans and Kep levels (*P* < 0.05), but not with Ve and *P* > 0.05 levels. Magnetic resonance imaging can be used to diagnose prostate cancer. It can differentiate and diagnose different types of prostate cancer early. This is important for evaluating the benefits of prostate cancer screening and treatment.

## 1. Introduction

Prostate cancer is a very common cancer in the male. It is mainly caused by the elderly and is a highly malignant reproductive system. The incidence rate of this disease is very high, which is next only to gastric cancer. With the development of aging society in recent years, the incidence rate and mortality of prostate cancer are increasing year by year [1]. Therefore, it is the key factor to ensure the rehabilitation of patients and guide various treatment plans by using appropriate regimen to diagnose patients. Magnetic resonance diffusion-weighted imaging is a very common clinical diagnostic scheme (see Figure 1); it mainly uses an image comparison formed by the difference of internal or local magnetic sensitivity in the magnetic field as the diagnostic scheme. The imaging basis of this diagnostic scheme is mainly high-resolution and three-dimensional complete flow compensated gradient echo sequence, which can clearly show the patient's intracranial lesions [2].

Prostate cancer mostly occurs in elderly men over the age of 60, and the periphery of the prostate is a frequent area of the disease. This disease will have a great impact on the normal life of elderly men, and most elderly patients will have a more serious psychological adverse state after the onset, which will have a great adverse impact on the normal life of elderly patients. In the traditional diagnostic scheme, patients are usually diagnosed by ultrasound or CT, but the diagnostic accuracy is often low. Puncture biopsy is an open diagnostic scheme, which has a certain adverse impact on patients. At the same time, elderly patients are often combined with patients with other systemic and organic diseases, which is not only painful but also prone to transfer and implant with the puncture needle path [3]. Dynamic enhanced scanning can clarify the cancerous tissue and microvessel status of patients to a certain extent. Because the vascular density in cancerous tissue is higher than that in normal tissue and is evenly distributed, the application of enhanced scanning can clarify the changes of cancerous tissue by observing vascular proliferation. Diffusion-weighted MRI has a good clinical diagnostic effect. This diagnostic scheme can diagnose the diffusion movement of water molecules in tissues. It is also the only diagnostic scheme that can play this effect in clinic. Generally speaking, water molecules often have high degrees of freedom when diffusing in the human body, which belongs to diffusion type movement, and will be limited when the surrounding tissues change, which is called diffusion limitation. Diffusion-weighted MRI can effectively diagnose the diffusion degree and direction of water molecules and further reflect the microstructure of the tissue. When the patient's tissue is cancerous, the patient's normal tissue will be excluded and banned by cancerous tissue, and the water molecular weight contained in it will be reduced. Therefore, in this case, the content of water molecules in cancerous tissues will decrease, and cancerous tissues tend to be distorted and narrow in the process of proliferation. Therefore, diffusion-weighted can effectively clarify the cancer status and prostate tissue changes of patients in this situation, and this scheme belongs to noninvasive diagnosis scheme, which will not cause additional adverse effects on patients and has high diagnostic significance. According to the clinical stage obtained by MRI and the GS score obtained by the pathological results of biopsy tissue, the condition of patients with PCA can be evaluated comprehensively and accurately [4]. Some studies have shown that the preoperative pathological grading of prostate cancer plays a very important guiding role in clinical diagnosis and treatment, such as the low-risk cancer in the low-risk group with GS score ≤ 6. Clinically, local treatment and dynamic observation can often be adopted, and some inert cancer foci may be carried for life without any progress. Those with Gleason score > 6 are medium- and high-risk cancers, which need scientific and correct intervention and treatment. Therefore, blind treatment or overtreatment of some patients in clinic cannot achieve the expected effect and even cause serious adverse effects. It can be seen that early accurate diagnosis of PCA patients and accurate risk classification have important guiding significance for the treatment and prognosis of patients [5].

## 2. Literature Review

Seo et al. believe that magnetic resonance imaging (MRI) can provide important evidence for the clinical diagnosis, staging, and treatment of prostate cancer because of its high resolution of soft tissue and the advantages of multiparameter, multisequence, and multidirectional imaging. At present, it is considered to be one of the most ideal examination methods in the examination of prostate diseases. With the upgrading of magnetic resonance imaging equipment, the improvement of technology, and the enrichment of functional imaging methods, magnetic resonance imaging can provide more basis for the diagnosis and classification of prostate cancer and provide important evidence for the selection of clinical diagnosis and treatment of prostate cancer [6]. The proposal of pi-rads V2 in Trufanov et al. is mainly to diagnose prostate cancer according to the advantages of different sequences on different anatomical sites and tissue structures. High-resolution T2WI was the main diagnosis of cancer lesions in the central gland area; DWI sequence and ADC image are the main reference for the diagnosis of peripheral diseases; DCE sequence was used when the benign and malignant lesions could not be determined (the score was 3 points). In the junction area between the central area and the peripheral zone, T2WI is mainly used. When the benign and malignant cannot be determined, DWI sequence is supplemented [7]. Peeters et al. believe that according to the clinical stage obtained by MRI and the GS score obtained by the pathological results of biopsy tissue, the condition of patients with PCA can be evaluated comprehensively and accurately [8]. Conte et al. proposed that the preoperative pathological grading of prostate cancer plays a very important guiding role in clinical diagnosis and treatment. For example, for low-risk cancer in low-risk group with GS score ≤ 6, local treatment and dynamic observation can often be adopted clinically, and some inert cancer foci may be carried for life without any progress. Those with Gleason score > 6 are medium- and high-risk cancers, which need scientific and correct intervention and treatment [9]. The research of Antunes et al. shows that multiparameter magnetic resonance imaging (MP MRI) can provide more accurate and rich diagnostic information that is helpful to clinic. Other studies have shown that T2WI combined with magnetic resonance functional imaging sequences greater than or equal to two can significantly improve the sensitivity and specificity of image examination for PCA diagnosis and then improve the diagnostic efficiency [10]. Yildirim first used apt imaging technology to detect free proteins and amino acids in vivo in 2003. Under the principle of proton saturation and proton free exchange with water, the proton can be detected indirectly under the principle of proton saturation and proton free exchange with water [11]. Pinto et al. proposed that all prostate cancers (CHO + CRE)/CIT ≥ 0.86. In the peripheral zone of prostate, when its value ≥0.75, it may be cancer [12]. Pecherkin et al. proposed that the diagnostic standard of prostate cancer in Chinese is >0.99 [13]. Eichhoff et al. proposed that the diagnostic standard of prostate cancer in Chinese is >1.09/0.94 (before all/D stage), but when the cancer focus is small and limited, taking 0.94 as the standard has greater diagnostic significance. However, MRS is easily affected by the internal environment, and its parameters are prone to deviation. In the presence of inflammation, hyperplasia, and partial volume effect, its specificity and sensitivity are reduced. In matrix based gland hyperplasia, its metabolic characteristics are similar to those of prostate cancer, and its value overlaps to a certain extent, so it cannot be well identified [14].

Based on the current research, prostate cancer (PCA) is one of the common malignant tumors in elderly men. With the aggravation of China's aging population and the continuous improvement of examination technology, the detection rate of prostate cancer has a significant upward trend. Magnetic resonance imaging technology is an imaging examination method that has emerged in recent years. It occupies an important position in clinical examination with the advantages of high-resolution, multiplanar parameter imaging, and no radiation. At present, it has become the first choice for noninvasive diagnosis of prostate cancer. With the progress of imaging, the emergence of magnetic sensitivity-weighted imaging (SWI) further provides a reliable way for clinical diagnosis of diseases. It uses different magnetic sensitivities between different tissues to detect the distribution of blood vessels and mineral deposits in the lesions. This study examined SWI in patients with different types of early prostate cancer and benign prostatic hyperplasia in our hospital to explore the clinical diagnostic value of SWI in different types of early prostate cancer. The report is as follows.

## 3. Data and Methods

### 3.1. General Information

60 patients with prostate cancer treated in 2019 were selected as the study group. All patients were tested for prostate-specific antigen (PSA). They were divided into different groups according to the range of PSA value, of which 0-4 mg/ml was group A (*n* = 18), 5-10 mg/ml was group B (*n* = 26), and > 10 mg/ml was divided into group C (*n* = 16). Procedures include (1) division and focal hypotension around the prostate; (2) MRI routine (T1WI, T2WI, DCE, and SWI); (3) patients have been diagnosed with prostate cancer through surgery, infection, or a blood test; (4) no relationship between diagnosis and treatment before MRI. Procedures: prost prostate cancer; and (5) before prostatectomy, the prostate needs to be biopsied. At this time, more than 60 patients with prostate hyperplasia who were admitted to our hospital were selected for the panel. The mean age of the patients in this study was 34-65 years, on average (49.6 ± 5.2). Patients on the control group were 60-66 years of age and of median age (50.2 ± 5.4). There were no significant differences between the two groups (*P* > 0.05) in the above data (sex and age).

### 3.2. Method

1. SWI examination methods: the patients were examined by magnetic resonance sensitivity-weighted imaging with Siemens1.5TSkyra magnetic resonance scanner. The patient took the supine position and took the 2.0 cm above the pubic symphysis as the scanning center for the axial, sagittal, and coronal TSET2WI sequence scanning of the prostate [15]: TR 6500 ms, TE 104 ms, layer spacing 0 mm, layer thickness 3 mm, matrix384 × 607, average 2, and FOV180mm × 180 mm. SWI scanning parameters are as follows: TR 28 ms, TE 20 ms, turning angle 150, FOV 180 mm × 180 mm, layer thickness 3 mm, matrix 384 × 365, automatic generation of amplitude image, phase image, SWI image, and minimum density projection (MIP) image. After the second dynamic phase of dynamic contrast-enhanced scanning, the contrast agent GD DTPA was injected through elbow vein with high-pressure syringe at the injection rate of 2 ml/s and the dose of 0.2 mmol/kg, and then, 20 ml normal saline was injected intravenously at the same rate [16]
2. Image analysis method SWI image processing and analysis: two senior doctors in the imaging department of our hospital jointly evaluate the film. Their opinions are not unified at one time, and a unified opinion is reached through negotiation [17]. According to the SWI image obtained by the patient, the internal bleeding focus of the focus was evaluated by SUSE score. SUSE scoring standard is as follows: 0: no bleeding; 1 point: there are 1-5 points and linear bleeding foci; 2 points: there are 6~10 points and thread mounted bleeding foci; and 3 points: more than 10 point and linear bleeding foci [18].

### 3.3. Observation Indicators

The levels of SUSE score, transport constant (Ktrans), extracellular space volume percentage (Kep), and rate constant (Ve) were observed, and the relationship between SUSE and the levels of Ktrans, Kep, and Ve in patients with prostate cancer was analyzed [19].

### 3.4. Statistical Treatment

SPSS18.0 statistical software was used. The counting data was expressed in percentage, *x*^2^ test was used, and the measurement data was expressed in $\overset{¯}{x}\pm s$, and *t* test was used. The comparison between multiple groups was analyzed by analysis of variance, *F*-value test, and Spearman's analysis. *P* < 0.05 was the difference with statistical significance [20].

## 4. Experimental Results and Analysis

### 4.1. Comparison of SUSE Score and Ktrans, Kep, and Ve Levels in Each Group

There was no Ve phase difference between the four groups (*P* > 0.05); SUSE scores, Ktrans, and Kep were higher than group B, group B was higher than group A, and group A was higher (see Figure 2). The difference was significant (*P* < 0.05) (see Figures 3–6) [21].

### 4.2. Relationship between SUSE Score and Ktrans, Kep, and VE Levels in Patients with Early Prostate Cancer

SUSE score was positively correlated with the levels of Ktrans and Kep in patients with early prostate cancer (*P* < 0.05). There was no correlation with Ve level, *P* > 0.05 (see Figure 7) [22].

### 4.3. Discussion

Prostate cancer is one of the common malignant tumors in men. With the aging of China's population, the detection rate of prostate cancer is higher and higher, with an obvious upward trend. Magnetic sensitivity-weighted imaging (SWI) is a technique in magnetic resonance imaging [23]. At present, it is used in the examination of various malignant tumors and is widely used in clinic. SWI mainly quantifies the difference through the difference of magnetic sensitivity between different tissues and reflects the variables of tissue characteristics. It is examined by high-resolution, three-dimensional complete flow compensated gradient echo sequence. In recent years, it has been found in the study of prostate cancer that the microvessel density and vascular growth factor level of prostate cancer tissue are significantly higher than those of benign prostate tumors, neovascularization is more prone to bleeding, and a large amount of deoxyhemoglobin can increase magnetic sensitivity [24]. Benign tumors are inflammatory reactions, which only cause accelerated blood flow, relatively complete blood vessel wall, and low magnetic sensitivity. Therefore, some scholars believe that SWI scanning plays an important role in differentiating prostate cancer and benign prostate tumor. SWI examination of patients with prostate cancer and benign prostatic hyperplasia in our hospital showed that SUSE score and Ktrans and Kep levels were different in patients with different types of prostate cancer. SUSE score and Ktrans and Kep levels in group C were higher than those in group B, group B was higher than that in group A, and group A was higher than that in the control group. Ktrans can reflect the important index of the diffusion rate of contrast agent from intravascular to extraluminal. Kep is an index reflecting the rate of contrast medium flowing back from the extracellular space to the lumen. In the results of this study, the levels of Ktrans and Kep in group C were the highest. Studies have shown that due to the relatively large number of neovascularization and incomplete vascular endothelial cells in malignant tumors, the contrast medium exudes faster during contrast examination. The results suggest that malignant tumor cells grow vigorously and have more neovascularization, and the vascular basement membrane is incomplete. Therefore, the contrast agent is easy to penetrate outside the blood vessel, and the penetration speed is faster. Similarly, the reflux speed of contrast agent from the extravascular space to the blood vessel is also significantly faster. Therefore, the levels of Ktrans and Kep in group C are higher. Benign tumor tissue has less neovascularization, relatively complete vascular endothelium, and relatively slow penetration and reflux of contrast medium. The degree of malignant transformation in group A and group B was lower than that in group C, so the levels of Ktrans and Kep were lower than those in group C. Ve is the volume ratio of extravascular cell space to the whole voxel, which mainly reflects the percentage of contrast agent staying in extravascular cell space. The results showed that there was no difference in VE Levels among the four groups, which may be due to the simultaneous increase of Ktrans and Kep levels in groups A, B, and C, Ve = Ktrans/Kep, so the Ve value was relatively stable. SUSE score is an index reflecting the bleeding focus of prostate diseases. The higher the malignant degree of malignant tumor cells, the more prone to bleeding. Therefore, SUSE score in group C is significantly higher than that in other groups and the lowest in the control group. When observing the relationship between SUSE score and Ktrans and Kep levels, it was found that SUSE score was significantly positively correlated with Ktrans and Kep levels. Therefore, the higher the SUSE score, the higher the Ktrans and Kep levels, and the higher the malignancy of prostate cancer [25, 26].

## 5. Conclusion

In conclusion, when diagnosing prostate cancer patients, the application of magnetic sensitive diffusion-weighted imaging can effectively identify the specific symptoms of patients. However, the type of diagnosis needs to be selected according to the specific disease of the patient. If necessary, it also needs to select a variety of diagnosis schemes or carry out diagnosis for many times in combination with the specific clinical symptoms of the patient. This is of positive significance for the rehabilitation of patients and is worthy of popularization and use.

## Figures and Tables

**Figure 1:** MRI susceptibility-weighted imaging scanning diagnosis.

**Figure 2:** Comparison of SUSE scores and Ktrans, Kep, and Ve levels in each group of patients.

**Figure 3:** Comparison of SUSE score and Ktrans, Kep, and Ve levels of patients in group A.

**Figure 4:** Comparison of SUSE score and Ktrans, Kep, and Ve levels in group B patients.

**Figure 5:** Comparison of SUSE score and Ktrans, Kep, and Ve levels of patients in group C.

**Figure 6:** Comparison of SUSE score and Ktrans, Kep, and Ve levels in the control group.

**Figure 7:** Comparison of SUSE scores and Ktrans, Kep, and Ve in each group of patients.

## Data Availability

The data used to support the findings of this study are available from the corresponding author upon request.
